This article has been retracted.

# ECT2 Increases the stability of EGFR and Tumorigenicity by Inhibiting Grb2 Ubiquitination in Pancreatic Cancer

**DOI:** 10.3389/fonc.2020.589241

**Published:** 2021-02-08

**Authors:** Junxiong Wang, Shuo Yang, Li Min, Shengtao Zhu, Shuilong Guo, Shutian Zhang

**Affiliations:** ^1^Department of Gastroenterology, Beijing Friendship Hospital, Capital Medical University, Beijing, China; ^2^Beijing Key Laboratory for Precancerous Lesion of Digestive Diseases, Beijing, China; ^3^National Clinical Research Centre for Digestive Diseases, Beijing, China; ^4^Department of Laboratory Medicine, Peking University Third Hospital, Beijing, China

**Keywords:** PDAC, ECT2, EGFR, Grb2, EMT, ubiquitination

## Abstract

The poor prognosis of patients with pancreatic ductal adenocarcinoma (PDAC) is associated with the invasion and metastasis of tumor cells. Epithelial cell transforming 2 (ECT2) is a guanine nucleotide exchange factor (GEF) of the Rho family of GTPases. It has also been reported that upregulation of ECT2 in pancreatic cancer, but the role and mechanism of ECT2 have not been previously determined. We found that ECT2 was significantly elevated in PDAC tissues and cells, correlated with more advanced AJCC stage, distant metastases, and overall survival of patients with PDAC. Inhibition and overexpression tests showed that ECT2 promoted proliferation, migration and invasion *in vitro*, and promoted tumor growth and metastasis *in vivo*. We determined that ECT2 was involved in the post-translational regulation of Grb2. ECT2 inhibited the degradation of Grb2 through deubiquitination. Furthermore, knockdown of ECT2 downregulated EGFR levels by accelerating EGFR degradation. EGF stimulation facilitated the formation of ECT2-Grb2 complex. Overall, our findings indicated that ECT2 could be used as a promising new therapeutic candidate for PDAC.

## Introduction

ECT2 is located on the human chromosome 3q26.1-q26.2. As a guanine nucleotide exchange factor (GEF) of the Rho family of GTPases (1), ECT2 protein plays an important role in cell division (2). Rho family GTPases are involved in a variety of tumor progression signaling pathways (3). It has also been reported that upregulation of ECT2 in prostate cancer (4) and colorectal cancer (5) promotes malignant progression and predicts poor prognosis. Moreover, high expression level of ECT2 was associated with poor overall survival for pancreatic cancer patients (6). However, the role and mechanism of ECT2 in pancreatic cancer still remain unknown.

EGFR plays a critical role in the progression of pancreatic cancer, which is overexpressed in pancreatic cancer (7). The high expression of EGFR is closely related to the tumor metastasis and poor prognosis of patients with pancreatic cancer (7, 8). Under EGF stimulation, downstream signaling pathways activate and regulate cell proliferation, migration and survival (8). Growth factor receptor-bound protein 2 (Grb2) is an adaptor protein widely expressed in many cells by regulating the receptor tyrosine kinase (RTK) signaling pathway. Grb2 recognizes and binds phosphorylated EGFR through SH2 domain and two SH3 domains (9–11). Grb2 recruits the E3 ubiquitin ligase Cbl, resulting in ubiquitination of the EGFR and EGFR degradation. Interaction with the GTP-bound active form of Ras results in Raf activation and initiation of the MAPK signaling cascade (12, 13).

In the present study, we investigated the expression and clinical significance in PDAC cells and primary tumors. Furthermore, we found that ECT2 promoted proliferation, migration, and invasion *in vitro* and tumor metastasis *in vivo* by Ubiquitinating Grb2 protein. Knockdown of ECT2 decreased the EGFR and induced MET. EGF stimulation promotes the formation of ECT2-Grb2 complex. Our research reveals a previously unknown mechanism of ECT2 in the progression of PDAC, in which ECT2 up-regulates Grb2 expression, leading to tumor growth and metastasis.

## Materials and Methods

### Ethics Statement

Our research is conducted in accordance with the Declaration of Helsinki and international standards. All patients obtained written informed consent for this study, and the research protocol and process have been approved by the clinical research ethics committee of Beijing Friendship Hospital, Capital Medical University.

### Data Sources and Bioinformatics

Oncomine and The Cancer Genome Atlas (TCGA) were used for predictive bioinformatics data. In Oncomine database, we retrieved the “ECT2” and selected the differential gene analysis (pancreatic cancer and normal) to obtain differential expression results. TCGA-PAAD-RNA-Seq dataset was downloaded from TCGA database, which included 178 PDAC tissues and four adjacent normal tissues (14).

### Cell Culture and Transfection

Five pancreatic cancer cell lines (AsPC1, BxPC3, CAPAN, PANC1, and SW1990) and human pancreatic ductal epithelial cells hTERT-HPNE were purchased from the American Type Culture Collection (Manassas, VA). Cells for experiment were obtained from the original stock preserved in liquid nitrogen. All of the cancer cell lines were maintained in RPMI 1640 or DMEM Medium (Invitrogen) and supplemented with 10% fetal bovine serum (FBS), 100 U/ml penicillin, and 100 mg/ml streptomycin (Invitrogen, Shanghai, China) at 37°C with 5% CO2. Specially, HPNE cell was cultured as described (15).

Plasmid of pLKO.1-shECT2, pLKO.1-shGrb2, ECT2-Flag, Grb2-Flag, and Scramble clone vectors were purchased from GENECHEM (Shanghai, China). Lentivirus was prepared following the instructions. The cells were subcultured to 10% confluence in a medium containing puromycin (Sigma-Aldrich, St. Louis, MO, USA). Antibiotic-resistant clones were picked and passed in medium containing puromycin. The level of expression was assessed by Western blot assay.

### Western Blotting and Immunofluorescence

Cell lysate was prepared in RIPA buffer with addition of protease inhibitor cocktail, phosphatase inhibitor cocktail, DTT (Dithiothreitol), and Benzonase (Sigma-Aldrich, St. Louis, MO, USA). Protein concentration was calculated by the BCA Protein assay kit (Thermo Scientific Pierce, UK). Western blotting was performed using a standard method.

Antibodies for ECT2,Grb2, EGFR, AKT, pAKT, E-cadhein, N-cadhein, and Vimentin were purchased from Cell Signaling Technology Inc. (Beverly, MA). Antibody against actin was purchased from Santa Cruz Biotechnology (Santa Cruz, CA).

For immunofluorescence, briefly, cells were seeded on coverslips in six-well plates and fixed with 4% paraformaldehyde (PFA) at room temperature for 10 min. After three PBS-T (PBS with 0.1% tween-20) washes, cells were blocked first 5% BSA in PBS-T, then with Image-It @FX Signal Enhancer Ready Probes Reagent (Life Technologies). The cells were incubated with primary antibody overnight at 4°C and then incubated with Alexa Fluor^®^ 594 goat anti-rabbit or Alexa Fluor^®^ 488 goat anti-mouse (Molecular Probes). The slides were counterstained with DAPI and imaged using the confocal laser-scanning microscope LSM510 Meta (Carl Zeiss).

### TMA and Immunohistochemistry

The study included a total of 100 PDAC patients, 80 of whom had adjacent normal tissues. The operation was performed from September 2004 to December 2008, and the patient was followed up until October 2012 or died. The median follow-up time was 12 months (range 0.6–87 months). During the follow-up period, 71 patients died of PDAC. All operations were R0 resection. The age, gender, pathological grade, TNM staging (according to AJCC), family history, smoking history, drinking history and type II diabetes history were collected. There was no significant difference in baseline characteristics between PDAC patients and adjacent normal tissue (control group) patients (**Supplementary Table 1**).

Immunohistochemistry (IHC) for ECT2 and Grb2 protein expression in TMA was performed by standard methods. The tissue sections were deparaffinized and hydrated. 3% H_2_O_2_ was used to block the endogenous peroxidase activity. 0.01M citrate buffer (pH 6.0) and microwave heat induction were used for antigen retrieval. ECT2 staining was scored according to the percentage and intensity of positive cells. The staining intensity was scored in four levels: 0 (no staining), 1 (weak staining), 2 (medium staining) and 3 (strong staining).

### *In Vitro* Migration, Invasion, and Wound Healing Assays

Migration and invasion assays were carried out in 24-well plates using Boyden chambers with an 8-mm pore size PET membrane (Falcon). Briefly, cells were transfected with ECT2 or Grb2 shRNA; Cells was counted and processed for transwell assay. After a night, each of non-invasive cells on the upper surface of the Matrigel membrane was gently removed. The invasive cells were fixed with anhydrous methanol and stained with toluidine blue. Under an inverted optical microscope, the stained cells that have passed through the membrane surface were photographed and quantified in three randomly selected areas. Results were obtained from three independent experiments performed in duplicate.

The wound healing assay was done by using ECT2 shRNA or non-specific shRNA cells. Briefly, when cells were grown to confluent, we used the 100 μl tip to scratch in the middle of the well. After this, we took photos of different wound regions and the size of the wound was calculated by image-J software (NIH, USA) and the relative wound closure was analyzed.

### Soft Agar Colony Formation Assay

The cells were seeded in six-well plates containing agar. Growth medium with 10% FBS was added to the top of the agar. The cell suspension was plated and cultured in a 37°C incubator for 14 days. Finally, the colonies were fixed with 4% PFA, stained with crystal violet and counted.

### *In Vivo* Xenograft Model

The animals were kept in facilities approved by the Animal Protection Committee of Capital Medical University, and experiments are carried out in accordance with the animal experiment guidelines. Tumor cells were injected into the axilla to establish subcutaneous tumor formation, and tail vein injection was used to establish a lung metastasis model.

Nude mice (BALB/c-nu) were acclimatized for a week. Stably transfected ASPC-1 cells (5×10^6^) were resuspended in PBS and implanted into axilla of male BALB/c nude mice by subcutaneous injection. The difference between tumor sizes of shScramble- and shECT2-transfected groups (12 mice per group) was evaluated. After the mice were sacrificed, the tumor tissues were excised and the weight and volume were measured. Finally, samples were extracted for various tests.

AsPC-1 cells (1 × 10^7^/ml) suspended in 100μl FBS-free medium were injected into the tail veins of 10 nude mice. The mice were sacrificed after 6 weeks. The number of lung metastases was counted, and then HE staining.

### Immunoprecipitaion

The protein G Dynabeads were pre-washed and incubated with rabbit anti-ECT2, mouse anti-Grb2, or their rabbit or mouse IgG control antibodies in 5% BSA IP buffer for 6 h. And then the beads were washed with IP buffer five times on a magnet. ASPC-1 cells were grown to a density of 70%–90% in a 15 cm dish, and then lysed with IP buffer for 30 min on ice. Lysates were cleared by centrifugation. Add 2 mg of total protein to the beads and incubated at 4°C for 2 h. After that, the beads were washed six times. Finally, boil the protein on the beads with 1x protein SDS, and boil it on a heating block at 95°C for 10 min. Immunoprecipitates were analyzed using SDS-PAGE.

### Statistical Analysis

Experimental data are presented as the mean ± standard deviation (SD). Statistical analyses were performed using analysis of a two-tailed Student’s t test or chi-square test with either GraphPad Prism 5 (GraphPad Software, Inc., La Jolla, CA, USA) or SPSS Statistics software (version 20.0, Chicago, Ill). Survival curves were calculated using the Kaplan-Meier method. Differences were considered statistically significant when P values were less than 0.05.

## Results

### High Expression of ECT2 Is Associated With More Aggressive Clinicopathological Features of PDAC Patients

In order to clarify the function of ECT2 in pancreatic cancer, we first evaluated the expression of ECT2 in the pancreatic cancer datasets of Pei Pancreas. We found that the mean expression value of ECT2 was significantly increased in PDAC tissues compared with the adjacent normal tissues (**Figure 1A**). To identify the expression of ECT2 in pancreatic cancer, we have analyzed 40 pairs of PDAC and normal tissues adjacent to cancer. ECT2 expression was significantly upregulated in tumor samples compared to normal tissues (*P*<0.001; **Figure 1B**). The expression of ECT2 was further tested by IHC in the TMA containing 80 paired PDAC tissues (**Figure 1C**). The correlation of ECT2 enhancement with clinicopathological features of pancreatic cancer patients was then explored. Patients were divided into low-ECT2 group and high-ECT2 group. We revealed a positive association between ECT2 overexpression and advanced histological grade, advanced AJCC stage, tumor size, distant metastases, smoking and Type II diabetes (**Table 1**). However, no significant association was observed between ECT2 expression with gender, age or lymph node metastasis. We found that high ECT2 expression was correlated significantly with poorer survival (**Figure 1D**). In addition, Pearson’s correlation test in the TCGA_PAAD dataset showed that ECT2 was positively correlated with Ki-67 (r = 0.7939, p <0.0001, n = 178) (**Figure 1E**).

**Figure 1:** High expression of epithelial cell transforming 2 (ECT2) is associated with more aggressive clinicopathological features of pancreatic ductal adenocarcinoma (PDAC) patients. **(A)** Increased expression of ECT2 mRNA in pancreatic adenocarcinoma compared to normal pancreas in Pei Pancreas dataset (GEO: GSE 16515). **(B)** RT-PCR analysis of ECT2 gene expression in PTAC and normal tissue adjacent to cancer. **(C)** Representative TMA immunohistochemistry (IHC) images of ECT2 in PDAC tissues and normal pancreatic tissue. Scale bars: 500 *µ*m (left), 200 *μ*m (middle), and 400 *μ*m (right). **(D)** Patients with higher ECT2 expression displays worse OS (*p*=0.0108) compared to ECT2-low group. **(E)** TCGA_PAAD dataset showed ECT2 was positively correlated with Ki-67(r=0.7939, p < 0.0001, n=178) in PDAC tissues. *p < 0.05.

**Table 1:** Association between epithelial cell transforming 2 (ECT2) expression and the clinicpathological features of PDCA.

Characteristics	Number	ECT2 expression		*P* value
		High (n=45)	Low (n=55)	
Age(years)				
<60	50	21	29	0.99
≥60	50	24	26	
Gender				
Male	62	31	31	0.22
Female	38	14	28	
Pathology grade				
I-II	78	27	51	**0.007**
above II	22	15	7	
Vessel/nerve invasion				
Yes	43	19	24	1.00
No	57	26	31	
Tumor invasion depth				
T1,T2	79	40	39	0.08
T3,T4	21	5	16	
Lymph node metastasis				
N0	58	26	32	0.97
N1	42	19	23	
Distant metastasis				
M0	96	41	55	**0.02**
M1	4	4	0	
AJCC-stage				
I-II	74	28	46	**0.04**
above II	26	17	9	
Tumor size				
<5cm	60	20	40	**0.007**
≥5cm	40	25	15	
Smoking status				
Yes	36	24	12	**0.002**
No	64	21	43	
Type II diabetes				
Yes	32	23	9	**<0,001**
No	68	22	46	

Bold values indicate statistical differences.

### ECT2 Promoted PDAC Cells Colony and Proliferation *In Vitro*

PANC-1, AsPC-1, and CAPAN-1 cell lines were chosen for further investigation because of their high or low expression of ECT2 (**Figure 2A**). To investigate whether ECT2 positively regulates cell colony and proliferation, we employed the shRNA targeting ECT2 in PANC-1, AsPC-1 cells and established stable overexpression of ECT2 in CAPAN-1 cell. The transfection efficiency was confirmed by qRT-PCR. Firstly, the colony of shECT2 transfection group was significantly less than that of NC group (**Figure 2B**). Simultaneously, CAPAN-1/ECT2 cells had significantly more colonies compared with their control cells (**Figure 2C**). These results were further confirmed by cell proliferation assay. Knockdown of ECT2 expression significantly attenuated the growth of PANC-1 and AsPC-1cells (**Figures 2D, E**). Overexpression of ECT2 significantly promotes the growth of CAPAN-1 cells (**Figure 2F**), indicating that ECT2 promotes PDAC growth.

**Figure 2:** Epithelial cell transforming 2 (ECT2) promoted pancreatic ductal adenocarcinoma (PDAC) cells colony and proliferation *in vitro*. **(A)** The expression of ECT2 in HPNE cell lines and PDAC cell lines. **(B)** Use effective shRNAs to knockdown ECT2, transfection efficiency was measured by qRT-PCR. The number of colonies of PANC-1 cells transfected with shRNA targeting ECT2 was significantly less than that of the NC group. **(C)** Colony numbers of PANC-1 cells transfected with ECT2-Flag were significantly more than numbers of NC groups. **(D, E)** CCK-8 assay showed knockdown of ECT2 inhibited both AsPC-1 and PANC-1 cells proliferation. **(F)** CCK-8 assay showed ECT2 overexpress promoted CAPAN-1 cells proliferation. *p<0.05, **p<0.01.

### Loss of ECT2 Inhibits Cell Migration, Invasion, and EMT *In Vitro*

We further investigated the role of ECT2 in the progression of PDAC. ECT2 knockdown significantly inhibited migration and invasion of PDAC (*p <*0.001; **Figure 3A**). Overexpression of ECT2 can significantly enhance the migration and invasion of PDAC (*p <*0.001; **Figure 3B**). Moreover, the wound healing assay also showed that the migration ability of ECT2 knockdown cells was significantly reduced compared to normal cells (*p <*0.05; **Figure 3C**). In addition, PANC-1 cells grew as scattering distribution and, upon ECT2 knockdown, acquired a circular shape and compact colonies, suggesting Mesenchymal epithelial transformation phenomenon (**Figure 3D**).

**Figure 3:** Loss of ECT2 inhibits cell migration, invasion and EMT *in vitro*. **(A)** Representative pictures show the effect of epithelial cell transforming 2 (ECT2) shRNA treatment on cell migration and invasion. Scale bar: 100 *μ*m. **(B)** Representative pictures show the effect of ECT2-Flag treatment on cell migration and invasion. Scale bar: 100 *μ*m. **(C)** Representative images of wound healing assay show the effect of stable knockdown of ECT2 on HCC cell migration. **(D)** Phase contrast microphotographs of AsPC-1 cells infected with either shNC or ECT2-targeting shRNA. Scale bar: 100 *μ*m. Three independent experiments were performed for cell migration and invasion assays and wound healing assays, respectively.

### ECT2 Exerts Its Malignant Activity *via* Influencing Grb2

We revealed that ECT2 promoted proliferation and metastasis in pancreatic cancer. On the mentha website, through “protein-protein interaction analysis and prediction”, it was found that there is a protein interaction between ECT2 and Grb2 (**Figure 4A**). Further, we found that knockdown of ECT2 lead to inhibition of Grb2 and phosphorylation of Akt. Simultaneously E-cadherin increased, Vimentin and N-cadherin reduced (**Figure 4B**). It was suggested that ECT2 may regulate EMT *via* Grb2/Akt pathway. As shown in **Figure 4C**, in immunohistochemistry for ECT2 and Grb2 protein, ECT2 expression was also significantly positively correlated with Grb2 expression (p<0.01, n=100). Immunofluorescence showed that Grb2 was highly expressed in the negative control group, while it was significantly reduced in the shECT2 group (**Figure 4D**). Our results indicated that ECT2 might promote the proliferation and metastasis of PDAC cells by partially regulating Grb2.

**Figure 4:** Epithelial cell transforming 2 (ECT2) exerts its malignant activity *via* influencing Grb2. **(A)** Protein prediction map for interaction with ECT2, from mentha website. **(B)** Western blot validated Grb2 protein and downstream signaling was markedly affected in ECT2-KD group. The activity of Grb2 downstream signaling molecules and EMT-relative markers were analyzed by immunoblotting. β-actin was used as a loading control. **(C)** In Immunohistochemistry results, Grb2 was positively correlated with ECT2 expression(r=0.5068, p<0.01, n=100). **(D)** Immunofluorescence staining showed that pancreatic ductal adenocarcinoma (PDAC) cell lines infected with ECT2-targeting shRNA expressed low levels of Grb2. The nucleus was stained with 40, 6-diamidino-2- phenylindole in the merged images. Scale bar: 100 *μ*m.

### ECT2 Interacts With Grb2 Leading to Its Deubiquitination

We found that Grb2 level was decreased in the shECT2 cells compared with NC. Co-IP analysis was used to verify the potential interaction between ECT2 and Grb2 in PANC-1 cells. Endogenous ECT2 was found to be associated with Grb2 and conversely endogenous Grb2 was found to be immunoprecipitated with ECT2 (**Figure 5A**). ECT2 interacting with Grb2 confirmed the specificity of their interaction. In addition, ubiquitination assay confirmed that the loss of ECT2 significantly increased the level of Grb2 ubiquitination, thereby protecting Grb2 from degradation. The proteasome inhibitor cycloheximide (CHX) was used to block protein degradation, and the interaction between ECT2 and GRB2 led to GRB2 deubiquitination (**Figure 5B**).

**Figure 5:** Epithelial cell transforming 2 (ECT2) interacts with Grb2 leading to its deubiquitination. **(A)** Endogenous ECT2 and Grbs were immunoprecipitated under denaturing conditions from PANC-1 cells. **(B)** The cell lysates of the control and ECT2 knockdown ASPC-1 cells were immunoprecipitated with anti-Grb2 antibody, and the immunocomplexes were immunoblotted with anti-Grb2 and anti-ubiquitin antibodies in the presence of cycloheximide(CHX). **(C)** Molecules in stable PANC-1 cells with ECT2 or Grb2 knockdown were determined by the western blot. **(D)** The ASPC-1 cells were treated with EGF in the presence of cycloheximide (CHX). The cell lysates were then immunoprecipitated with anti-EGFR antibody, and the immunocomplexes were immunoblotted with anti-Grb2 and anti-ECT2 antibodies. **(E, F)** Knocking down ECT2 reduces EGFR and baseline phosphorylation levels of ERK and Akt and also decreases the level of maximal phosphorylation of ERK and Akt. *p < 0.05.

Previously, it was reported that Grb2 can promote EGFR endocytosis and intracellular transport, thereby inhibiting EGFR degradation and leading to the termination of signal transduction (13). Therefore, we investigated whether ECT2 regulated EGFR by Grb2 in pancreatic cancer cells. To determine whether Grb2 is required for ECT2-mediated EGFR regulation, we measured Grb2 in PANC-1 cell silencing of ECT2. Downregulation of ECT2 resulted in reduction of EGFR and Grb2. Knockdown of Grb2 inhibited the expression of ERFR and the activation of downstream pathways. We detected that ECT2 silencing inhibited EGFR signaling pathway and downstream targets E-cadherin. Then this inhibitory effect was amplified when cells were pretreated with Grb2 loss (**Figure 5C**), indicating that the interaction between ECT2 and Grb2 leads to increased EGFR and promotes EMT of pancreatic cancer cells. Endogenous ECT2 interacts with Grb2, while EGF stimulation can promote the formation of ECT2-Grb2 complex (**Figure 5D**). Grb2 induced EGF receptor protein accumulation. When PANC-1 cells were pretreated with EGF in the presence of cycloheximide, we found the degradation of EGFR in the ECT2 knockdown group was significantly faster than that in the control group. ECT2 silencing significantly inhibited EGF function, including inhibiting the increase of the key proteins in EGF/EGFR-ERK/Akt signaling (pAkt and pERK)(**Figure 5E**). We quantified the results of Western Blot in **Figure 5F**. It indicated that the ECT2 could regulate the degradation of EGFR and downstream signaling pathways.

### ECT2 Promotes Cancer Progression Through Grb2

We further verified whether ECT2 regulates the process of PDAC in a Grb2-dependent manner. Grb2 was down-regulated in PDAC cells. The knockdown efficiency was verified by western blot (**Figure 6A**). Colony formation and CCK-8 assays showed that the reduction of Grb2 significantly inhibited tumor cell proliferation (**Figures 6B, C**).In addition, we rescued the expression of Grb2 in ECT2 silenced PDAC cells. Interestingly, the overexpression of Grb2 can partially attenuate the inhibition of Akt activation and EMT marker vimentin mediated by ECT2 silence (**Figure 6D**). The restoration of Grb2 expression eliminated the inhibition of ECT2 depletion-induced proliferation and invasion abilities (**Figures 6E, F**). Taken together, these findings indicated that ECT2 regulates the progress of PDAC upstream of Grb2.

**Figure 6:** Epithelial cell transforming 2 (ECT2) promotes cancer progression through Grb2. **(A)** PANC-1 and ASPC-1 cells were treated with shRNAs targeting Grb2. The knockdown efficacy was measured by western blot. **(B)** Proliferation of pancreatic ductal adenocarcinoma (PDAC) cells was detected by CCK-8 assay. **(C)** Colony formation assay was also used to detect the proliferation of PDAC cells. **(D)** Western blot analysis was used to verify the rescue effect of Grb2 on ECT2 knockdown. **(E)** Grb2 abolished the proliferation inhibition induced by ECT2 knockdown in PANC-1 cells as confirmed by CCK-8 assays. **(F)** GRB2 abolished the invasion inhibition induced by ECT2 knockdown in the PANC-1 cells as confirmed by the transwell assays. *p < 0.05.

### Inhibition of ECT2 Suppresses Tumor Growth and Metastasis *In Vivo*

The roles of ECT2 in pancreatic cancer cells *in vitro* were further verified using *in vivo* mice models. ECT2-silenced AsPC-1 cells were subcutaneously injected into the nude mice. Compared with NC group, the ECT2-depleted group revealed significant reductions in tumor size (**Figure 7A**), tumor volume and weight (**Figures 7B, C**).

**Figure 7:** Inhibition of epithelial cell transforming 2 (ECT2) suppresses tumor growth and metastasis *in vivo*. **(A)** Xenograft model in nude mice and harvested nodules from NC group and ECT2-KD group. **(B, C)** Tumor nodules derived from sh-ECT2-transfected cells are significantly smaller and lighter than those in NC group. **(D)** Western blot validated Grb2 protein was markedly decreased in ECT2-KD group. EGFR/Akt/ERK signaling pathway and EMT-relative markers were analyzed by immunoblotting. β-actin was used as a loading control. **(E)** Downregulation of ECT2 significantly suppressed lung metastasis of pancreatic ductal adenocarcinoma (PDAC) cells. Scale bar: 200 *μ*m. *p<0.05, **p<0.01.

Western blotting showed that decreased levels of Vimentin, N-cadherin decreased and E-cadherin increased accompanied by inhibition of EGFR/Akt/ERK pathways in ECT2 knockdown group compared to the negative control groups (**Figure 7D**).

To explore the effects of ECT2 on lung metastasis of PDAC cells, ECT2-silenced AsPC-1 cells were injected in the tail vein of nude mice. The mice were sacrificed 6 weeks later. The lung tissue was H&E stained after consecutive section. The number of lung metastases was independently calculated and evaluated by two pathologists. As shown in **Figure 7E**, the rate of lung metastasis was lower in ECT2 knockdown group than in negative control groups. The data indicated that ECT2 depletion represses the growth and metastasis of pancreatic cancer cells *in vivo*.

## Discussion

ECT2 is reported to be upregulated in several types of cancer (16, 17). Chen J et al. (18) found that ECT2 activated Rho/ERK signal to promote early recurrence in human hepatocellular carcinoma. Wang Y et al. (19) found that PKC1 binded to ECT2 *via* Par6 to form a complex and activates the MEK-ERK signaling pathway in ovarian cancer. Justilien et al. (20) reported that ECT2 was required for lung tumorigenesis and that Rac1 and PKC1 mediated ECT2 phosphorylation to promote ribosomal RNA (rRNA) synthesis. The prognosis of PDAC remains dismal and our knowledge of the underlying cellular molecular pathways remains limited. In this study, our results demonstrated ECT2 was significantly overexpressed in PDAC tumors. In addition, it was found that the up-regulation of ECT2 expression predicted a shorter overall survival time for PDAC patients. We further demonstrated that ECT2 played critical roles in the proliferation, migration and invasion of PDAC cells, and promotes the growth and metastasis of tumors *in vivo*.

The GEF ECT2 has multiple substrates, including Rac1, RhoA, and Cdc42 (21). Here, we demonstrate that ECT2 is a positive regulator of Grb2 in pancreatic cancer. Grb2 plays a key role in enhancing the malignant characteristics of cancer cells (22), and that ubiquitination of Grb2 is still elusive. We revealed the potential mechanism of Grb2 regulation mediated by ECT2. We found that Grb2 protein levels and its downstream signaling were suppressed by ECT2 knockdown. The loss of ECT2 accelerated the degradation of Grb2 protein. In addition, Grb2 ubiquitination was significantly increased due to ECT2 depletion. It has been previously reported that E6AP enhanced ECT2 ubiquitination and proteasome degradation (23). Interestingly, ECT2 can also affect the stability of E2F1 by regulating the expression of deubiquitinating enzyme PSMD14 (24). So the mechanism by which ECT2 regulates the ubiquitination of Grb2 remains to be further studied.

EGFR plays key roles in essential cellular functions, including proliferation and migration (13). Overexpression of EGFR occurs in >90% of pancreatic cancer and is associated with a poorer prognosis (25). EGFR signaling in pancreatic cancer promotes proliferation and invasion of pancreatic cancer by regulating EMT (26). Genetic studies in mice indicate that the development of PDAC requires EGFR expression. In the presence of oncogenic K-RAS mutants, EGFR plays an important role in acinar to ductal metaplasia (27, 28). In line with PDAC models, a kinase inhibitor specific to EGFR can sensitize tumors to chemotherapy (gemcitabine) (29). Indeed, EGFR inhibitors have shown limited but reproducible responses in PDAC patients, leading to US Food and Drug Administration approval of erlotinib for treating PDAC (Moore et al., 2007). A study confirmed that the combination of EGFR inhibitors and K-RAS-related inhibitors was a more effective way to treat PDAC (30).

In this study, knockdown of ECT2 decreased EGFR expression and inhibited its downstream signaling pathway. EGFR overexpresses in tumor tissue for two main reasons, one is gene amplification, and the other is blocked protein degradation. The data presented here suggested that ECT2 may potentially affect multiple cellular processes that drive PDAC progression through EGFR levels. ECT2 may regulate the level of Grb2 ubiquitination, while Grb2 ubiquitination reduces EGFR degradation. It is possible that the effect of ECT2 on EGFR may be mediated by Grb2.

Through the analysis of clinical data, we found that the high expression of ECT2 was related to advanced histological grade, advanced AJCC stage, distant metastases, smoking and Type II diabetes. At the same time, we observed a positive correlation between ECT2 and Grb2 and a poor prognosis for patients with high ECT2–expressing tumors. Therefore, our clinical data confirmed that ECT2 could promote the progression and metastasis of pancreatic cancer.

In conclusion, we have confirmed that ECT2 plays a key role in the progression of pancreatic cancer. These findings have important implications for the prognosis and treatment of PDAC. The expression level of ECT2 may represent a biomarker of EMT, which can predict invasiveness and metastasis. Drugs that inhibit the activity of ECT2 may block the downstream pathways of EGFR. This targeted therapy may be an effective method to inhibit Grb2. In summary, for the first time, we report the relation between ECT2 and Grb2 in pancreatic cancer metastasis. We demonstrate that high ECT2 expression in pancreatic cancer suppresses the ubiquitination of Grb2 and activates the EGFR signaling pathway to promote metastasis (**Figure 8**). Our findings highlight the ECT2-Grb2-EGFR axis as a potential target for therapeutic intervention in pancreatic cancer metastasis.

**Figure 8:** Upregulation of epithelial cell transforming 2 (ECT2) activates EGFR signaling *via* GRB2 deubiquitination and promote metastasis.

## Data Availability Statement

The datasets presented in this study can be found in online repositories. The names of the repository/repositories and accession number(s) can be found in the article/**Supplementary Material**.

## Ethics Statement

The animal study was reviewed and approved by Ethics Committee of Beijing Friendship Hospital. Written informed consent was obtained from the individual(s) for the publication of any potentially identifiable images or data included in this article.

## Author Contributions

JW and SZhang conceived and contributed to design of the study. SY and LM performed the experiments. SZhu and SG analyzed and interpreted the data. JW and SZhang supervised and contributed to writing the manuscript. All authors contributed to the article and approved the submitted version.

## Funding

This research was supported by Capital Medical University Research and Development Fund (PYZ2017149, PYZ2018151), Digestive Medical Coordinated Development Center of Beijing Municipal Administration of Hospitals (XXT05). The funding sponsors had no role in the design of the study; in the collection, analyses, or interpretation of data; in the writing of the manuscript, and in the decision to publish the results.

## Conflict of Interest

The authors declare that the research was conducted in the absence of any commercial or financial relationships that could be construed as a potential conflict of interest.

## Abbreviations

AJCC, American Joint Committee on Cancer; DAPI, 4’,6-diamidino-2-phenylindole; ECT2, epithelial cell transforming 2; EGFR, epidermal growth factor receptor; EMT, epithelial mesenchymal transition; FBS, fetal bovine serum; GEF, guanine nucleotide exchange factor; IHC, immunohistochemistry; PDAC, pancreatic ductal adenocarcinoma; TCGA, The Cancer Genome Atlas; TMA, tissue microarray.
